The article "NEAT1 Overexpression Indicates a Poor Prognosis and Induces Chemotherapy Resistance via the miR-491-5p/SOX3 Signaling Pathway in Ovarian Cancer" was retracted in 2022. Reasons: original data or images not available; concerns about the data.

# NEAT1 Overexpression Indicates a Poor Prognosis and Induces Chemotherapy Resistance via the miR-491-5p/*SOX3* Signaling Pathway in Ovarian Cancer

**DOI:** 10.3389/fgene.2021.616220

**Published:** 2021-04-29

**Authors:** Xinzhuan Jia, Lan Wei, Zhengmao Zhang

**Affiliations:** ^1^Department of Reproductive Medicine, The Fourth Hospital, Hebei Medical University, Shijiazhuang, China; ^2^Department of Chest Surgery, Hebei Chest Hospital, Shijiazhuang, China; ^3^Department of Gynecology, The Fourth Hospital, Hebei Medical University, Shijiazhuang, China

**Keywords:** NEAT1, miR-491-5p, *SOX3*, exosomes, ovarian cancer, chemoresistance

## Abstract

**Background:**

Accumulated studies have reported that dysregulated long non-coding RNAs (lncRNAs) are crucial in ovarian cancer (OC) initiation and development. However, detailed biological functions of lncRNA NEAT1 during the progression of OC remains to be uncovered.

**Purpose:**

Our aim was to identify the role of NEAT1 in cisplatin resistance of ovarian cancer and the underlying mechanisms.

**Methods:**

The expression patterns of NEAT1 in OC cell lines and tissue samples were identified by qRT-PCR. The cisplatin (DDP) sensitivity of OC cells was detected by MTT and CCK8 assay, while OC cell apoptosis and cell cycle were detected using flow cytometer assays. In addition, effects of NEAT1 on tumor growth were determined by xenograft tumor model. Luciferase reporter assay was conducted to prove the regulatory relation of miR-491-5p, NEAT1, and *SOX3*. Importantly, the expression of NEAT1 in exosomes from cisplatin-resistant patients was also determined by using qRT-PCR.

**Results:**

In this study, upregulated NEAT1 was detected in OC cell lines and tissues. Meanwhile, NEAT1 was also increased in cisplatin-resistant OC cell lines and tissues. Upregulation of NEAT1 inhibited cisplatin-induced OC cell apoptosis and promoted cell proliferation, while knockdown of NEAT1 played the opposite role. These effects were also observed *in vivo*. Furthermore, direct interaction was observed between NEAT1 and miR-491-5p. NEAT1 led to the upregulation of miR-491-5p-targeted *SOX3* mRNA. Importantly, this study also showed upregulated NEAT1 expression in serum exosomes derived from cisplatin-resistant patients.

**Conclusion:**

NEAT1 is vital in the chemoresistance of ovarian cancer through regulating miR-491-5p/*SOX3* pathway, showing that NEAT1 might be a potential target for OC resistance treatment.

## Introduction

Ovarian cancer (OC), as one of gynecologic cancers with the highest mortality, accounts for 5% malignancies in female patients worldwide (Siegel et al., 2019). Although the aggressive surgical techniques developed in the past decades, the survival of OC patients has not been considerably improved (Yang et al., 2020). Chemotherapy is widely used for treating locally advanced and metastatic OC in clinical settings; however, chemoresistance is inevitable during the long course of treatment, with the 5 years survival rate of OC patients limited to 40% (Jiang et al., 2019). Due to lack of sensitive approaches for early diagnosis and the prevention of resistance to chemotherapy, most patients eventually succumb to recurrent, progressive cancers (Qiu et al., 2019; Yang Y. et al., 2019). In consequence, the prevention, diagnosis and treatment may benefit from deeper knowledge of molecular mechanisms involved in ovarian carcinogenesis.

The article "NEAT1 Overexpression Indicates a Poor Prognosis and Induces Chemotherapy Resistance via the miR-491-5p/SOX3 Signaling Pathway in Ovarian Cancer" was retracted in 2022. Reasons: original data or images not available; concerns about the data.

Long non-coding RNAs (lncRNAs), as a family of non-coding RNAs with over 200 nt, have now been considered important in multiple pathophysiologic processes, including proliferation, migration, invasion, metastasis, apoptosis, cell cycle, and drug resistance in in cancers (Shang et al., 2019; Yang H. et al., 2019). Hence, functional lncRNAs might be used as potential prognostic biomarkers and therapeutic targets. Mounting lncRNAs were determined to be dysregulated and were associated with the development and progression of OC (Zhang et al., 2018). In addition to the functions in cancer proliferation, lncRNAs also involved in cancer cell responses to the chemotherapy (Ren et al., 2018; Cai et al., 2019). For instance, upregulated SNHG22 indicated poor prognosis and induced chemotherapy resistance in epithelial ovarian carcinoma through the miR-2467/Gal-1 signaling pathway (Zhang et al., 2019). Meanwhile, regulatory mechanisms of lnc00161/miR-128/MAPK1 axis on drug resistance were also demonstrated in OC (Xu et al., 2019). It has been reported that NEAT1 is an oncogene in various cancers, such as bladder cancer (Shan et al., 2020), hepatocellular carcinoma (Krohler et al., 2019), prostate cancer (Jiang et al., 2020), non-small cell lung cancer (Qi et al., 2018). Previous studies have shown that NEAT1 is a candidate marker for the prediction of the invasiveness and prognosis of OC (Chen et al., 2016). Nevertheless, the roles and clinical significance of NEAT1 in cisplatin resistance of OC has not been identified. We hypothesized that NEAT1 could participant in the cisplatin-resistance of OC and the potential mechanism might be through miRNA modulation.

This study showed an increase of NEAT1 in cisplatin-resistant OC cell lines and tissues. Experiments also demonstrated the effect of NEAT1 on the sensitivity of OC cells to cisplatin. Our results create new insights that NEAT1 exerts critical roles in cisplatin resistance of OC by regulating the miR-491-5p/*SOX3* pathway.

The article "NEAT1 Overexpression Indicates a Poor Prognosis and Induces Chemotherapy Resistance via the miR-491-5p/SOX3 Signaling Pathway in Ovarian Cancer" was retracted in 2022. Reasons: original data or images not available; concerns about the data.

## Materials and Methods

### Patient Samples

OC tissues and the paired para-carcinoma tissues were collected from 90 primary OC patients from September 2010 to June 2015 at Department of Gynecology of The Fourth Hospital of Hebei Medical University. A chemotherapy-resistant case was distinguished when the primary tumor enlarged or relapsed within 6 months; otherwise, it can be defined as a chemotherapy-sensitive case. These tissue sample sections were immediately restored in liquid nitrogen for further study. The serum samples from these 90 patients were collected for exosome purification. Patients without preoperative treatments, including chemotherapy, radiotherapy or hormonal therapy were enrolled. This study was approved by the Research Ethics Committee of The Fourth Hospital of Hebei Medical University. Written informed consent forms were acquired from all subjects.

### Cell Culture and Treatment

Human OC cell lines (HO8910/DDP, HO8910, A2780, A2780/DDP, 3AO, SKOV3, CaoV-3) and normal human ovarian epithelial cell line CHO 1-15 from American Type Culture Collection (ATCC) were cultured in Dulbecco’s modified Eagle’s medium (DMEM; Invitrogen, Carlsbad, CA) containing 10% fetal bovine serum (Invitrogen) and penicillin/streptomycin (Invitrogen) in 5% CO_2_ at 37°C.

OC and OC resistant cells were collected at 70–80% cell confluence. Vector overexpressing NEAT1 was obtained from Sangon (Shanghai, China), while NEAT1 siRNAs and negative control siRNAs were acquired from GenePharma (Shanghai, China). The lentivirus vector containing small hairpin RNA (shRNA) sequence targeting NEAT1 (sh-NEAT1) was amplified and cloned by GenePharma (Shanghai, China). Moreover, miR-491-5p mimic, inhibitor and scrambled mimic control (miR-NC) were commercially acquired from RiboBio (Guangzhou, China) (Tan et al., 2019). The sequence of NEAT1 siRNA: 5′- GGAGGGCUAAUCUUCAACU-3′; negative control: 5′-AGGUAGUGUAAUCGCCUUGTT-3′; sh-NEAT1: 5′- TCAT GGACCGTGGTTTGTTACTATAGTGT-3′; sh-NC: 5′-CACCG TTCTCCGAACGTGTCACGTCAAGAGATTACGTGACACGT TCGGAGAATTTTTTG-3′. Lipofectamine 2000 reagent (Sangon) was used for the transfection of 35 nM siRNA (negative control siRNA as NC) or vector (empty vector as negative control, NC)in OC and OC resistant cells. Constructed sh-NEAT1 or sh-NC lentivirus was infected into cells, respectively. These cells were screened using puromycin for over 7 days to obtain stable NEAT1 knockdown cell line.

### Quantitative Real-Time PCR

Trizol reagent (Invitrogen, Carlsbad, CA, United States) was applied for extracting total RNAs from cells and tissues as per manufacturer’s protocol. Nanodrop spectrophotometer (ND-100; Thermo Scientific, Waltham, MA) was applied for the detection of RNA concentrations at 260/280nm absorbance. The expression levels of *GAPDH*, lnc-NEAT1 and *SOX3* were detected by SYBR Premix Ex Taq and TaqMan gene expression assays (Applied Biosystems, Foster City, CA, United States). In addition, miR-491-5p and U6 expressions were detected by Taqman Universal Master Mix II and TaqMan MicroRNA Reverse Transcription kit (Applied Biosystems). By using relative quantification as 2^–ΔΔ^CT, relative expressions were standardized and calculated to provide the fold change of gene expressions. The primers used were presented as below: NEAT1: 5′-CTTCCTCCCTT TAACTTATCCATTCAC-3′ (forward primer) and 5′-CTCTTCCTCCACCATTACCAACAATAC-3′ (reverse primer); miR-491-5p: 5′-GGAGTGGGGAACCCTTCC-3′ (forward primer) and 5′-GTGCAGGGTCCGAGGT-3′ (reverse primer); GAPDH: 5′-TATGATGATATCAAGAGGGTAGT-3′ (forward primer) and 5′-TGTATCCAAACTCATTGTCATAC-3′ (reverse primer); U6: 5′-CTCGCTTCGGCAGCACA-3′ (forward primer) and 5′-AACGCTTCACGAATTTGCGT-3′ (reverse primer); *SOX3*: 5′-GACCTGTTCGAGAGAACTCATCA-3′ (forward primer) and 5′-CGGGAAGGGTAGGCTTATCAA-3′ (reverse primer);

The article "NEAT1 Overexpression Indicates a Poor Prognosis and Induces Chemotherapy Resistance via the miR-491-5p/SOX3 Signaling Pathway in Ovarian Cancer" was retracted in 2022. Reasons: original data or images not available; concerns about the data.

### Western Blot

The total protein was obtained using RIPA (Beyotime, Shanghai, China) with Protease Inhibitor Cocktail (Roche, Basel, Switzerland), and protein concentrations were measured using a BCA Protein Assay Kit (Thermo Scientific Pierce). Proteins were segregated using SDS-PAGE, transferred onto PVDF membrane and blocked in 5% skim milk for 1 h at 37°C. Primary antibodies against *SOX3* (1:1,000, ab183606, Abcam) and GAPDH (1:1,000, ab181602, Abcam) were subject to overnight incubation onto the membrane at 4°C, followed by three runs of rinsing in TBST. After adding HRP-labeled goat anti-rabbit secondary antibody (1:2,000) into PVDF membrane, 1 h incubation was performed (Thermo Scientific). Enhanced chemiluminescence and Image J were used for the visualization and analysis of immunoreactive proteins, respectively.

### Flow Cytometry Analysis of Cell Apoptosis

Cells (2 × 10^5^ cells) were seeded into the six-well plates - and then were subjected to different transfections followed by diverse treatments (4 mg/mL of cisplatin or PBS). For cell apoptosis, the collected cells were rinsed twice in PBS. An Annexin V-FITC Apoptosis Detection Kit (BD Pharmingen, Mountain view, CA) was applied for cell apoptosis detection following its instructions. Cells re-suspended with 1X binding buffer were stained using Annexin V and PI away from light before flow cytometry analysis for 30 min (BD Biosciences, San Jose, CA, United States). The apoptotic cells were determined by a flow cytometer.

### CCK-8 Assay

Cell Counting Kit (Beyotime, Shanghai, China) was used for determining cell viability. In brief, cells were seeded into 96-well plates (5 × 10^3^ cells/well) and were subjected to specified treatments. After 72 h of incubation at 37°C, another 2 h of cell incubation with CCK-8 reagent was conducted. Multi-label plate reader (Bio-Rad, Hercules, CA, United States) was used for reading cell viability at 450nm.

The article "NEAT1 Overexpression Indicates a Poor Prognosis and Induces Chemotherapy Resistance via the miR-491-5p/SOX3 Signaling Pathway in Ovarian Cancer" was retracted in 2022. Reasons: original data or images not available; concerns about the data.

### Drug Resistance Assay

Drug resistance was determined using (4-5-dimethylthiazol-2-yl)-2,5-diphenyl tetrazolium bromide (MTT) assay. Before exposure to different doses of cisplatin, A2780, A2780/DDP, HO8910, HO8910/DDP cells were transfected with different agents for 24 h. After that, 20 μL of MTT (5 mg/mL, Sigma-Aldrich) was added into each well for another 4 h, and then 150 μL of DMSO was added for dissolving the formazan crystals. The absorbance was detected at 570 nm with a microplate reader. The relative survival curve was used for determining the cisplatin concentration that induced 50% cell growth inhibition (IC50).

### Luciferase Reporter Assay

Bioinformatics tools (Starbasev2.0 and TargetScan) were applied for the analysis of miR-491-5p binding sites on NEAT1 gene and *SOX3* binding sites on miR-491-5p. NEAT1 or 3′UTR of *SOX3* sequences with mutant-type or wild-type miR-491-5p binding sites were subject to synthesis and clone into pGL3 luciferase vectors (Promega, Madison, WI, United States) to generate NEAT1-WT or *SOX3*-WT and NEAT1-MT or *SOX3*-MT reporter vectors. The sequence of these above genes was shown in Figures 4, 5. For NEAT1, 293 T cells were subject to co-transfection with NEAT1-WT or NEAT1-MT and miR-491-5p or miR-con by Lipofectamine^TM^ 2000 (Invitrogen). For *SOX3*, *SOX3*-WT or *SOX3*-MT was transfected into 293 T with miR-con, miR-491-5p, miR-491-5p + Vector or miR-491-5p + pcDNA-NEAT1. Cells were collected at 48 h post transfection, with the luciferase activity measured by Dual Luciferase Reporter Assay Kit (Promega, Madison, WI, United States) following its instructions.

### Xenograft Tumor Model

BALB/c-nude female mice (4–5 weeks old, 18–20g) were procured from Shanghai Experiment Animal Centre, Shangai, China) and housed in specific conditions. All the experimental procedures were approved by The Fourth Hospital of Hebei Medical University. HO8910 cells (2 × 10^6^) transfected with sh-NEAT1 or sh-NC were subcutaneously injected into the flank of all mice. 15 days later, the nude mice were intraperitoneally injected with 4 mg/kg DDP or PBS every 4 days. Width (W) and length (L) of the tumor were measured using calipers to calculate tumor volumes at 7, 11, 15, 19, 23, 27, and 31 days. The tumor volumes were calculated as (L^∗^W^2^)/2. Mice were intraperitoneally injected with 3% pentobarbital sodium and were sacrificed by excessive anesthesia with a dose of 90 ml/kg, and the tumors were collected for the follow-up study. The above steps were operated by reference to the guideline of the Institutional Animal Care and Research Advisory Committee of Hebei Medical University (No. 2010101). Animal experiments were conducted under a SPF condition in Animal Laboratory at Hebei Medical University.

The article "NEAT1 Overexpression Indicates a Poor Prognosis and Induces Chemotherapy Resistance via the miR-491-5p/SOX3 Signaling Pathway in Ovarian Cancer" was retracted in 2022. Reasons: original data or images not available; concerns about the data.

### Immunohistochemistry (IHC)

IHC analysis was carried out as previously detailed described (Zhou et al., 2020a). The primary antibody against Ki67 (Abcam, ab15580) was used. The expressions were evaluated according to the percentage of positive cells.

### Exosome Purification

The extraction of exosomes from serum specimens was performed using ExoQuick precipitation kit (SBI, System Biosciences, Mountain View, CA) following previous descriptions (Takahashi et al., 2019). The characterization of vesicles floated in PBS was conducted using electron microscopy and western blot.

### Statistical Analyses

All data were represented as mean ± SD. Statistical significance was determined according to *p*-values generated by Kruskal-Wallis or two-way ANOVA or unpaired two-tailed Student’s *t*-test. GraphPad Prism v6.2 (GraphPad Software) was used for statistical analysis.

## Results

### NEAT1 Was Upregulated in Cisplatin-Resistant OC

NEAT1 was previously reported to be increased in different cancers (Krohler et al., 2019; Jiang et al., 2020; Shan et al., 2020). We firstly examined its expression in OC tissues and the paired adjacent tissues. As a result, significantly up-regulated NEAT1 was identified in OC tissues (Figure 1A). Next, we investigated the relationship between NEAT1 expression and the clinicopathological characteristics of OC patients, as listed in Table 1. Additionally, NEAT1 expression was also increased in cisplatin-resistant OC tissues comparing to in cisplatin-sensitive OC tissues (Figure 1B). Meanwhile, patients with a higher NEAT1 expression displayed a lower overall survival rate than those with a lower NEAT1 expression (Figure 1C). We investigated whether there was also a dysregulated NEAT1 expression in OC cell lines (CaoV-3, 3AO, SKOV3, A2780, HO8910) compared with the normal human ovarian epithelial cell line (CHO 1-15), and found that NEAT1 was remarkably induced in OC cell lines, especially in HO8910 and A2780 cells (Figure 1D). We also used cisplatin-resistant cells to explore the altered expression pattern of NEAT1, and the results showed that there was an obvious enhancement of NEAT1 in both A2780/DDP and HO8910/DDP cells (Figure 1E), which indicated a role of NEAT1 in cisplatin-resistance of OC cells.

The article "NEAT1 Overexpression Indicates a Poor Prognosis and Induces Chemotherapy Resistance via the miR-491-5p/SOX3 Signaling Pathway in Ovarian Cancer" was retracted in 2022. Reasons: original data or images not available; concerns about the data.

**FIGURE 1:** NEAT1 was upregulated in cisplatin-resistant OC. **(A)** QRT-PCR analysis of NEAT1 expressions in OC or adjacent normal tissues. **(B)** Relative NEAT1 expression in cisplatin-resistant OC and cisplatin-sensitive OC. **(C)** Kaplan-Meier curve of the estimated overall survival of both low and high NEAT1 expression groups. **(D,E)** Relative NEAT1 expression in both cisplatin-resistant and cisplatin-sensitive OC cell lines. Data were reported as mean ± SD. *p < 0.05, **p < 0.01, ***p < 0.001.

**TABLE 1:** Correlation between NEAT1 and clinicopathological characteristics in OC patients.

Variable	NEAT1		*P*-value
	Low	High	
**Age (years)**			
≤50	21	20	>0.05
>50	24	25	
**FIGO stage**			
I–II	30	14	<0.05
III–IV	15	31	
**Grade**			
1	26	11	<0.05
2-3	19	34	
**Lymph nodes metastasis**			
Negative	25	16	<0.05
Positive	20	27	
**Chemotherapy**			
Sensitive	29	13	<0.05
Resistant	16	32	

### NEAT1 Affected the Proliferation and Apoptosis of OC Cells *in vitro*

Considering the dysregulated expression pattern of NEAT1 in OC cells, we further explored whether NEAT1 had a role in cisplatin resistance in OC. Thus, OC cells (HO8910 and A2780) were further transfected with NEAT1 overexpressed plasmid and cisplatin-resistant cells (HO8910/DDP and A2780/DDP) were transfected with NEAT1 siRNA. Transfection efficiency was assessed via qRT-PCR (Figure 2A). MTT assays were applied to estimate the effects of NEAT1 on cisplatin resistance. Our data indicated that NEAT1 down-expression sensitized both OC cells and cisplatin-resistant cells to cisplatin, whereas increased expression of NEAT1 showed induced cisplatin resistance (Figure 2B). Meanwhile, CCK-8 assay was also conducted for detecting the effects of NEAT1 on cell proliferation. It was implied that NEAT1 promoted proliferation of OC cells and silence of NEAT1 decreased proliferation of cisplatin-resistant OC cells (Figures 2C,D). Subsequently, flow cytometry analysis was also used for determining the effect of NEAT1 on cisplatin-induced apoptosis. It was suggested that NEAT1 overexpression decreased OC cell apoptosis and knock-down of NEAT1 induced apoptotic rate of cisplatin-resistant OC cells (Figures 2E–H).

**FIGURE 2:** NEAT1 affected the OC cell proliferation and apoptosis *in vitro.* **(A)** QRT-PCR analysis of NEAT1 expression in OC cells post transfection with si-NEAT1 or NEAT1 plasmid. **(B)** IC50 of cisplatin-resistant or cisplatin-sensitive cells with increased or decreased NEAT1 level. **(C)** Promotion effects of overexpressed NEAT1 on the proliferation of A2780 and HO8910 cells during CCK-8 assay. **(D)** Suppression of NEAT1 silencing on the proliferation of A2780/DDP and HO8910 cells with 4 mg/mL cisplatin as shown by CCK-8 assay. **(E–H)** Flow cytometry of apoptosis of A2780 and HO8910 cells post transfection with vector or pcDNA-NEAT1; A2780/DDP and HO8910/DDP cells post transfection si-Control or si-NEAT1 before the stimulation of 4 mg/mL cisplatin treatments. All tests were conducted for at least three times. Data were reported as mean ± SD. *p < 0.05, **p < 0.01, ***p < 0.001.

The article "NEAT1 Overexpression Indicates a Poor Prognosis and Induces Chemotherapy Resistance via the miR-491-5p/SOX3 Signaling Pathway in Ovarian Cancer" was retracted in 2022. Reasons: original data or images not available; concerns about the data.

### lncRNA NEAT1 Promoted Cisplatin Resistance *in vivo*

To identify the role of NEAT1 in cisplatin resistance *in vivo*, nude mice were subjected to HO8910 cells transfected with sh-NEAT1 or sh-NC. The results suggested that cisplatin treatment showed a remarkable inhibitory effect on tumor growth when compared to the control groups (Figure 3A). Additionally, after treating with cisplatin, mice with sh-NEAT1 injection displayed a smaller tumor volume and weight, which suggested that inhibition of NEAT1 repressed tumor cell resistance to cisplatin *in vivo* (Figures 3B,C). Correspondingly, compared to the control group, the number of tumor nodules was reduced by DDP or sh-NEAT1 treatment individually. The combination of the DDP and sh-NEAT1 further reduced the number and the size of the tumor nodules (Figure 3D). Moreover, immunohistochemistry assay of Ki-67 was also performed to verify the effects of NEAT1 on tumor cell proliferation, which suggested that downregulated NEAT1 had an inhibition on proliferation of tumor cells (Figure 3E). These results were consistent with the results *in vitro*, and further demonstrated that NEAT1 promoted cisplatin resistance *in vivo*.

**FIGURE 3:** lncRNA NEAT1 promoted cisplatin resistance *in vivo.* **(A)** Photos of tumors in xenograft-transplanted nude mouse tumor models after the treatment of oral cisplatin (qd) or NS as control for 31 days in different groups. **(B)** Measurements of tumor volumes every 4 days using calipers. **(C)** Weights of tumors in xenografts of different groups. **(D)** Representative images of the mesenteric membrane of six mice per group are shown. *Indicates tumor nodule. **(E)** IHC analysis of Ki-67 expression in xenografts of different groups. All tests were conducted for at least three times. Data were reported as mean ± SD. *p < 0.05, **p < 0.01, ***p < 0.001.

### NEAT1 Served as a Molecular Sponge of miR-491-5p in OC Cells

Accumulating evidences indicated that lncRNAs exerted their role via interacting with miRNAs (Xie et al., 2020; Zhou et al., 2020b). To determine the candidate target miRNAs of NEAT1, bioinformatic prediction analysis was performed by using Starbase online website. As a result, top 10 potential target miRNAs were detected, and miR-491-5p was identified as the target miRNA of NEAT1. Regulation of NEAT1 on miRNA expressions was then observed in OC cells (HO8910 and A2780) and cisplatin-resistant OC cells (HO8910/DDP and A2780/DDP). It was suggested that miR-491-5p expression was repressed after NEAT1 over-expression in HO8910 and A2780 cells, and silencing NEAT1 promoted miR-491-5p expression in HO8910/DDP and A2780/DDP cells (Figures 4A,B and Supplementary Figures S1A–D). We also detected miR-491-5p expression in OC tissues and cells. The results unveiled that miR-491-5p exhibited a lower expression in cisplatin-resistant OC tissues and OC cell lines (Figures 4C,D). Importantly, cisplatin-resistant cells also displayed a significantly decreased expression level of miR-491-5p compared with the corresponding OC cells. Regarding the ontogenetic roles of NEAT1 in cisplatin resistance in OC, the role of miR-491-5p in HO8910/DDP and A2780/DDP was also determined. Our data suggested that anti-miR-491-5p showed partial reversed effect of si-NEAT1-mediated anti-proliferation in HO8910/DDP and A2780/DDP cells (Figures 4E,F). To further identify the interaction of NEAT1 with miR-491-5p, luciferase reporter assay was conducted. Figure 4G displayed that miR-491-5p harbored a complementary binding sequence of NEAT1. Further experiments validated the interaction of NEAT1 with miR-491-5p. After transfecting with NEAT1-WT or NEAT1-MT luciferase reporter plasmids, the effects of NEAT1 on miR-491-5p were determined. We revealed that the luciferase activity of NEAT1-WT reporter systems was notably repressed post co-transfected with miR-491-5p mimic, suggesting that NEAT1 interacted with miR-491-5p through the putative binding site (Figures 4G,H). All the results signified that NEAT1 sponged miR-491-5p to repress its expression which further regulated the OC progression.

The article "NEAT1 Overexpression Indicates a Poor Prognosis and Induces Chemotherapy Resistance via the miR-491-5p/SOX3 Signaling Pathway in Ovarian Cancer" was retracted in 2022. Reasons: original data or images not available; concerns about the data.

**FIGURE 4:** NEAT1 functioned as a molecular sponge of miR-491-5p in OC cells. **(A)** Decrease in miR-491-5p expression by overexpressed NEAT1. **(B)** Increase in miR-491-5p expression by silencing NEAT1. **(C)** Relative miR-491-5p expression in cisplatin-sensitive and cisplatin-resistant OC groups. **(D)** Relative miR-491-5p expression in a set of OC cell lines. **(E,F)** Proliferation of si-NEAT1-treated cells decreased and rescued by miR-491-5p inhibitor during CCK8 assay. **(G)** Sequence of NEAT1 containing highly conserved putative miR-491-binding sites as shown by StarBase v.2.0. **(H)** Luciferase activity of NEAT1-WT luciferase reporter vector remarkably reduced by miR-491-5p mimic relative to NC. All tests were conducted for at least three times. Data were reported as mean ± SD. *p < 0.05, **p < 0.01, ***p < 0.001.

### *SOX3* Was a Direct Target of miR-491-5p

TargetScan online software was employed to further identify the underline mechanism of NEAT1/miR-491-5p axis on cisplatin resistance in OC cells. We found that *SOX3* was a target candidate of miR-491-5p (Figure 5A). For further verify the direct interaction of NEAT1 and miR-491-5p, the constructed *SOX3*-MT-3′UTR reporter systems and *SOX3*-WT-3′UTR luciferase reporter systems were co-transfected with miR-491-5p mimic or the negative control. These findings showed that transfection of miR-491-5p mimic tremendously inhibited the luciferase activity of *SOX3*-WT-3′UTR reporter systems in both HO8910 and A2780 cells (Figure 5B). As we expected, *SOX3* was notably decreased in cisplatin-resistant cell lines and tissues (Figures 5C,D). We further verified the regulation of NEAT1/miR-491-5p axis on *SOX3* as well. As shown in Figures 5E,F, miR-491-5p suppression notably reversed the downregulation of *SOX3* induced by NEAT1 inhibitor in HO8910/DDP and A2780/DDP cells (Figures 5E,F). To further verify the modulation of NEAT1 on OC cell proliferation and cell apoptosis through SOX3 axis, the si-SOX3 and NEAT1 overexpression plasmid were co-transfected into the HO8910/DDP and A2780/DDP cells. The results indicated that the suppressed proliferation and promoted apoptosis by si-SOX3 could be rescued by NEAT1 overexpression (Supplementary Figures S2A,B), which highly suggested that NEAT1 overexpression could induce chemotherapy resistance in ovarian cancer through the SOX3 signaling pathway.

**FIGURE 5:** SOX3 was a direct target of miR-491-5p. **(A)** Binding sites between SOX3 and miR-491-5p predicted by bioinformatics analysis. **(B)** Luciferase activity of SOX3-WT in OC cells considerably reduced by miR-491-5p mimics as indicated by luciferase reporter assay. **(C)** Relative SOX3 expression in OC patients. **(D)** Relative SOX3 expression in cancer cell lines. **(E,F)** Real-time PCR analysis and Western Blot assay for determining SOX3 expression in cells with rescue assay. All tests were conducted for at least three times. Data were reported as mean ± SD. *p < 0.05, **p < 0.01, ***p < 0.001.

### NEAT1 Was Secreted Into Exosomes From OC Patients’ Sera

Exosomes could prevent the degradation of lncRNAs in the circulation and transfer lncRNAs between cancer cells to transmit signals and phenotypes (Han et al., 2020). In this study, exosomes were extracted from serum samples of cisplatin-sensitive or cisplatin-resistant OC patients, and NEAT1 expression in exosomes of OC patients were defined. We characterized these vesicles by electron microscopy (Figure 6A) and western blot (Figure 6B). High expression levels of exosomal markers, such as TSG101 and CD63, were detected to verify the purity of OC-secreted exosomes in serum. This study also indicated that NEAT1 was highly expressed in serum samples of cisplatin-resistant patients compared to cisplatin-sensitive serum samples (Figure 6C). Moreover, a considerable inverse association was also identified between NEAT1 expression and miR-491-5p expression in exosomes in OC (Figure 6D). These results above indicated that NEAT1 in exosomes could be a potential diagnostic biomarker for cisplatin-resistant OC patients.

The article "NEAT1 Overexpression Indicates a Poor Prognosis and Induces Chemotherapy Resistance via the miR-491-5p/SOX3 Signaling Pathway in Ovarian Cancer" was retracted in 2022. Reasons: original data or images not available; concerns about the data.

**FIGURE 6:** NEAT1 was secreted into exosomes from OC patients’ sera. **(A)** Typical electron microscope image of exosomes from OC patients’ sera. **(B)** Western blotting for biomarkers of exosomes from purified serum exosomes. **(C)** QRT-PCR for the abundance of NEAT1 in serum exosomes, and NEAT1 levels in sera. **(D)** Negative association between NEAT1 and miR-491-5p expressions in exosomes extracted from OC patients’ sera. **p < 0.01.

## Discussion

Extensive clinical trial of conventionally PARP inhibitor (PARPi) therapies have shown that PARPis are particularly sensitive and effective against ovarian deficient in BRCA1, BRCA2, and PTEN DNA repair genes (Rose et al., 2020). However, cisplatin are still the current first-line drugs for ovarian cancer and other carcinomas for its effect on inducing DNA double-strand breaks (DSBs) and apoptosis of cancer cells (Mensah et al., 2019). Although chemotherapy is widely used for treating metastatic OC for the encouragingly efficiency, drug resistance remains to be a great challenge for its clinical use (Boyd and Muggia, 2018; Li et al., 2018; Sang et al., 2018; Jiang et al., 2019; Qu et al., 2019). In recent years, studies indicating that lncRNAs were associated with drug sensitivity of tumor cells have been increasingly concerned. For example, upregulated UCA1 was observed in the cisplatin-resistant tissues and cell lines, and UCA1 was reported to induce cisplatin resistance via the regulation of miR-143/FOSL2-signaling pathway in OC (Li Z. et al., 2019). The role of PANDAR in chemoresistance was verified in OC patients, and the possible mechanism might be related to its regulation of SFRS2-mediated p53 phosphorylation (Wang et al., 2018). LncRNA NEAT1 was demonstrated to enhance paclitaxel resistance of OC cells through the regulation of ZEB1 expression via miR-194 (An et al., 2017). HOTAIR was more abundant in the advanced OC tissues and was also overexpressed in cisplatin-resistant OC cell lines, compared to sensitive controls. Furthermore, HOTAIR expression was correlated with poor survival of patients who received carboplatin compared with the untreated patients (Wang et al., 2015). MALAT1 was demonstrated to correlate with NOTCH1 expression, which was also up-regulated during platinum resistance in OC (Bai et al., 2018). ZFAS1 overexpression was also identified to be one predictive marker of platinum-sensitivity, based on transcriptome data from 258 patients with HGSCs (Liu et al., 2017). Thus, more understanding of lncRNAs and the underlined mechanisms of lncRNAs might provide prospective the diagnostic and therapeutic options for OC.

The article "NEAT1 Overexpression Indicates a Poor Prognosis and Induces Chemotherapy Resistance via the miR-491-5p/SOX3 Signaling Pathway in Ovarian Cancer" was retracted in 2022. Reasons: original data or images not available; concerns about the data.

Recently, several studies identified that lncRNA NEAT1 was dysregulated and exerted its oncogenic roles in diverse tumors, such as breast cancer (Ghafouri-Fard and Taheri, 2019), non-small cell lung cancer (Qi et al., 2018), and colorectal cancer (Yu et al., 2019). Likewise, another study also revealed up-regulated NEAT1 in human OC cells compared to normal epithelial cells in OC, which was agreed with the previous study (Chen et al., 2016). Additionally, it was also indicated that NEAT1 might function as an oncogene in the pathogenesis of OC, which reported that NEAT1 enhanced cell migration and proliferation of OC cells (Li et al., 2016). Moreover, NEAT1 was also associated with paclitaxel resistance of OC cells (An et al., 2017). However, whether there is a function role of NEAT1 in cisplatin resistance in OC is still unclear. Here in our study, NEAT1 was also highly expressed in cisplatin-resistant OC tissues and cells. NEAT1 down-expression sensitized both OC cells and cisplatin-resistant cells to cisplatin, whereas increased NEAT1 induced cisplatin resistance, which indicated that NEAT1 might be a key factor in cisplatin resistance in OC.

Increasing evidences have indicated that lncRNAs exert their post-transcriptional roles as competing endogenous RNAs by sponging miRNA to exert their regulatory functions. In the recent years, studies have been conducted to show aberrant miRNA expressions in drug-resistant OC cells (Li J. et al., 2019). By using bioinformatics analysis (Starbase 2.0), miR-491-5p was predicted as a candidate target miRNA of NEAT1. miR-491-5p was determined to be downregulated in various cancers as a tumor suppressor by regulating its targeting genes as reported by the previous studies (Lu et al., 2019). For example, downregulated miR-491-5p enhanced metastasis of gastric cancer by regulating SNAIL and FGFR4 (Yu et al., 2018). miR-491-5p was also observed to induce apoptosis of OC cells by directly binding to BCL-XL and EGFR, which resulted in BIM activation (Denoyelle et al., 2014). Our study showed that miR-491-5p was considerably down-regulated in cisplatin-resistant OC tissues relative to cisplatin-sensitive OC tissues. Meanwhile, the anti-miR-491-5p showed partial rescued effects on si-NEAT1-mediated anti-proliferation in HO8910/DDP and A2780/DDP cells, indicating that NEAT1 sponges miR-491-5p which further regulates the OC progression. *SOX3*, as a member of SOX family transcription factors together with SOX1, SOX2, and SOX2, selectively interacts with the common target sequence and activates gene transcription 1 (Guo et al., 2018). In recent years, increasing evidences suggested the involvement of *SOX3* in tumorigenesis. *SOX3* was reported to act as an oncogene in different tumors, such as glioblastoma (Marjanovic et al., 2019) and esophageal squamous cell carcinoma (Li et al., 2013). In this study, *SOX3* was notably reduced in cisplatin-resistant cell lines and tissues. In further analysis, miR-491-5p regulated *SOX3* expression through directly targeting 3′ UTR of *SOX3*. Aberrant expression of miR-491-5p and *SOX3* in cisplatin-resistant OC may be a new therapeutic option for cisplatin resistance of OC patients.

The article "NEAT1 Overexpression Indicates a Poor Prognosis and Induces Chemotherapy Resistance via the miR-491-5p/SOX3 Signaling Pathway in Ovarian Cancer" was retracted in 2022. Reasons: original data or images not available; concerns about the data.

It is generally acknowledged that exosomes are implicated in drug resistance, tumor development and metastasis as a key component of tumor microenvironment (Tang et al., 2019), by carrying cancer-specific biomolecules shed from tumor cells. Furthermore, multiple exosomes were detected to be stably expressed in several body secretions (Chen et al., 2019), which makes exosomes and their specific biomolecules as stable non-invasive markers in the screening test, diagnosis examination and prognostic prediction of cancers. Additionally, exosomes detection regarding cancer detection, therapeutic effect assessment and prognostic prediction have been used in cancers such as non-small cell lung cancer (Liu et al., 2019). In the present study, NEAT1 was highly expressed in cisplatin-resistant serum exosomes relative to the cisplatin-sensitive serum exosomes, and it also showed an inverse correlation with miR-491-5p, indicating that NEAT1 and miR-491-5p in exosomes might be a promising biomarker for cisplatin-resistant OC.

## Conclusion

In conclusion, we identified up-regulated NEAT1 in OC and its role in cisplatin resistance of OC. Mechanistically, NEAT1 serves as a molecular sponge of miR-491-5p, which further targets *SOX3* to exert its functions in OC. These findings suggest us to deepen the understanding of functions and mechanisms of NEAT1 in cisplatin resistance in OC, and provide evidence that NEAT1 represents a potential diagnostic and therapeutic target for cisplatin-resistant OC.

## Data Availability Statement

The original contributions presented in the study are included in the article/Supplementary Material, further inquiries can be directed to the corresponding author/s.

The article "NEAT1 Overexpression Indicates a Poor Prognosis and Induces Chemotherapy Resistance via the miR-491-5p/SOX3 Signaling Pathway in Ovarian Cancer" was retracted in 2022. Reasons: original data or images not available; concerns about the data.

## Ethics Statement

The studies involving human participants were reviewed and approved by the Research Ethics Committee of The Fourth Hospital of Hebei Medical University. The patients/participants provided their written informed consent to participate in this study.

## Author Contributions

XJ made substantial contributions to conception and design. LW made acquisition of data and performed the experiments. XJ, LW, and ZZ wrote the draft manuscript. All authors contributed to the reviewing of the manuscript and approved the final manuscript for submission.

## Conflict of Interest

The authors declare that the research was conducted in the absence of any commercial or financial relationships that could be construed as a potential conflict of interest.

## Supplementary Material

Supplementary Figure 1 **(A,B)** HO8910/DDP and A2780/DDP cell lines treated with si-NEAT1 to detected the potential 9 miRNAs binding to NEAT1. **(C,D)** HO8910 and A2780 cell lines treated with NEAT1 overexpression plasmid to detected the potential 9 miRNAs binding to NEAT1. **(E)** HO8910 and A2780 cell lines treated with NEAT1-MUT and NEAT1-WT plasmid.

Supplementary Figure 2 A2780/DDP and HO8910/DDP were transfected by Control, si-SOX3, and si-SOX3 + NEAT1. **(A)** The proliferation of A2780/DDP and HO8910 cells were shown by CCK-8 assay. **(B)** Flow cytometry of apoptosis of A2780/DDP and HO8910 cells.
